The article "Territory-Wide Chinese Cohort of Long QT Syndrome: Random Survival Forest and Cox Analyses" was retracted in 2024. Reasons: lack of ethics approval or compliance; concerns about the welfare of human subjects.

# Territory-Wide Chinese Cohort of Long QT Syndrome: Random Survival Forest and Cox Analyses

**DOI:** 10.3389/fcvm.2021.608592

**Published:** 2021-02-05

**Authors:** Gary Tse, Sharen Lee, Jiandong Zhou, Tong Liu, Ian Chi Kei Wong, Chloe Mak, Ngai Shing Mok, Kamalan Jeevaratnam, Qingpeng Zhang, Shuk Han Cheng, Wing Tak Wong

**Affiliations:** ^1^Tianjin Key Laboratory of Ionic-Molecular Function of Cardiovascular Disease, Department of Cardiology, Tianjin Institute of Cardiology, Second Hospital of Tianjin Medical University, Tianjin, China; ^2^Faculty of Health and Medical Sciences, University of Surrey, Guildford, United Kingdom; ^3^Laboratory of Cardiovascular Physiology, Li Ka Shing Institute of Health Sciences, Hong Kong, China; ^4^School of Data Science, City University of Hong Kong, Hong Kong, China; ^5^Centre for Safe Medication Practice and Research, Department of Pharmacology and Pharmacy, Li Ka Shing Faculty of Medicine, The University of Hong Kong, Hong Kong, China; ^6^School of Pharmacy, University College London, London, United Kingdom; ^7^Department of Pathology, Hong Kong Children's Hospital, Hong Kong, China; ^8^Department of Medicine and Geriatrics, Princess Margaret Hospital, Hong Kong, China; ^9^Department of Biomedical Sciences, City University of Hong Kong, Hong Kong, China; ^10^State Key Laboratory of Agrobiotechnology, School of Life Sciences, Chinese University of Hong Kong, Hong Kong, China

**Keywords:** long QT syndrome, risk stratification, genetic variants, machine learning, random survival forest

## Abstract

**Introduction:** Congenital long QT syndrome (LQTS) is a cardiac ion channelopathy that predisposes affected individuals to spontaneous ventricular tachycardia/fibrillation (VT/VF) and sudden cardiac death (SCD). The main aims of the study were to: (1) provide a description of the local epidemiology of LQTS, (2) identify significant risk factors of ventricular arrhythmias in this cohort, and (3) compare the performance of traditional Cox regression with that of random survival forests.

**Methods:** This was a territory-wide retrospective cohort study of patients diagnosed with congenital LQTS between 1997 and 2019. The primary outcome was spontaneous VT/VF.

**Results:** This study included 121 patients [median age of initial presentation: 20 (interquartile range: 8–44) years, 62% female] with a median follow-up of 88 (51–143) months. Genetic analysis identified novel mutations in KCNQ1, KCNH2, SCN5A, ANK2, CACNA1C, CAV3, and AKAP9. During follow-up, 23 patients developed VT/VF. Univariate Cox regression analysis revealed that age [hazard ratio (HR): 1.02 (1.01–1.04), *P* = 0.007; optimum cut-off: 19 years], presentation with syncope [HR: 3.86 (1.43–10.42), *P* = 0.008] or VT/VF [HR: 3.68 (1.62–8.37), *P* = 0.002] and the presence of PVCs [HR: 2.89 (1.22–6.83), *P* = 0.015] were significant predictors of spontaneous VT/VF. Only initial presentation with syncope remained significant after multivariate adjustment [HR: 3.58 (1.32–9.71), *P* = 0.011]. Random survival forest (RSF) model provided significant improvement in prediction performance over Cox regression (precision: 0.80 vs. 0.69; recall: 0.79 vs. 0.68; AUC: 0.77 vs. 0.68; c-statistic: 0.79 vs. 0.67). Decision rules were generated by RSF model to predict VT/VF post-diagnosis.

The article "Territory-Wide Chinese Cohort of Long QT Syndrome: Random Survival Forest and Cox Analyses" was retracted in 2024. Reasons: lack of ethics approval or compliance; concerns about the welfare of human subjects.

**Conclusions:** Effective risk stratification in congenital LQTS can be achieved by clinical history, electrocardiographic indices, and different investigation results, irrespective of underlying genetic defects. A machine learning approach using RSF can improve risk prediction over traditional Cox regression models.

## Introduction

Long QT syndrome (LQTS) is characterized by an abnormally long QT interval on the electrocardiogram, which predisposes affected individuals to life-threatening ventricular tachycardia/fibrillation (VT/VF) and sudden cardiac death (SCD). They can result from a decrease in repolarizing currents or an increase in depolarizing currents at the cellular level and can have either congenital or acquired causes. Today, more than 16 genetic subtypes of congenital LQTS have been described. However, the overall aggregate risk of arrhythmogenesis depends on not only the genotypes but also on interacting clinical risk factors, leading to difficulty in accurate risk stratification.

The clinical and genetic epidemiology of congenital LQTS has been described in detail in Western populations. For example, differences in electrocardiographic variables have been observed between LQTS types 1, 2, and 3 (1). Bradycardia is a common feature regardless of subtype (1) and early-onset atrial fibrillation may be present (2). In Asia, several large-scale studies have been conducted in Japan. It was recently reported that pathogenic variants affecting the pore-forming regions of the ion channels led to more arrhythmic phenotypes within a particular LQTS subtype, and that gender-specific differences are seen in LQTS types 1 and 2, but not type 3 (3). However, the epidemiological and genetic data in Chinese patients are much less well-defined. A single-center study of 58 Chinese pediatric patients with congenital LQTS described the clinical course, confirming the presence of other arrhythmias such as sinus node dysfunction, atrioventricular block and atrial tachy-arrhythmias in addition to VT/VF (4). It also reported that LQTS type 3 was the most common, followed by Jervell and Lange-Nielsen syndrome type 1, LQTS types 1, 8, 2, and 4. The main aims of this territory-wide study from Hong Kong are (1) to provide a description of the local epidemiology of LQTS, (2) to identify significant risk factors of ventricular arrhythmias in this cohort, and (3) to compare the performance of traditional Cox regression with that of random survival forests. In doing so, we describe several novel genetic mutations that have not been previously identified in cohorts from other geographical regions.

The article "Territory-Wide Chinese Cohort of Long QT Syndrome: Random Survival Forest and Cox Analyses" was retracted in 2024. Reasons: lack of ethics approval or compliance; concerns about the welfare of human subjects.

## Methods

### Study Population

This retrospective study was approved by The Joint Chinese University of Hong Kong – New Territories East Cluster Clinical Research Ethics Committee (study approval number: 2019.338). The relevant datasets have been made available in an online repository. The inclusion criteria were patients diagnosed with congenital LQTS between 1997 and 2019 identified from searching the electronic health records from the Hospital Authority of Hong Kong. This system was previously used by our team to study other ion channelopathies such as Brugada syndrome (5, 6). Congenital LQTS was diagnosed if any of the following criteria were met: (i) Schwartz LQTS score ≥3.5, (ii) an unequivocally pathogenic mutation in one of the LQTS genes, (iii) corrected QT interval of ≥500 ms on repeated 12-lead ECG in the absence of a secondary cause for QT prolongation, in accordance with the 2013 Heart Rhythm Society Expert Consensus Statement (7). Those with unclassified variants were also included in the present analysis if there is a high clinical suspicion of LQTS or if prior clinical or functional studies have reported an arrhythmogenic phenotype.

### Extraction of Clinical and Electrocardiographic Data

Clinical data of included patients were extracted from their electronic health records. The following baseline clinical data were collected: (1) sex; (2) presentation age; (3) follow-up period defined as the time between presenting date and the date of last follow-up or death, whichever was earlier; (4) family history of LQTS and VT/VF/SCD; (5) initial presentation with syncope or spontaneous VT/VF, (6) development of syncope or VT/VF on follow-up and the number of episodes, if any; (7) electrophysiological study (EPS), 24-h Holter study, genetic testing and results; (8) performance of treadmill test and their effects on QTc prolongation on recovery, if present; (9) concomitant presence of other cardiac arrhythmias; (10) implantable-converter defibrillator (ICD) insertion; and (11) dosage regimen on the prescription of beta-adrenergic blockers and mexiletine.

Automatically measured parameters from baseline ECGs were extracted, including (1) heart rate; (2) P-wave duration; (3) PR interval; (4) QRS duration; (5) QT and QTc interval; (6) P-wave, QRS and T-wave axis; (7) S-wave amplitude in lead V1 and (8) R-wave amplitude in lead V5.

The article "Territory-Wide Chinese Cohort of Long QT Syndrome: Random Survival Forest and Cox Analyses" was retracted in 2024. Reasons: lack of ethics approval or compliance; concerns about the welfare of human subjects.

### Statistical and Survival Analyses

All statistical analysis was performed using Stata MP (Version 13.0). Categorical variables were expressed as total number (percentages). Continuous variables were expressed as mean ± standard deviation. The primary outcome of this study was spontaneous VT/VF. The above clinical and ECG variables were analyzed as risk factors for survival analysis. Cox regression with Efron's method for ties was used to identify independent predictors for shorter time to the first post-diagnosis VT/VF event. Variables achieving *P*-value < 0.10 were entered into multivariate analysis. Duration from the date of initial LQTS presentation to the first post-diagnosis VT/VF event for patient subgroups was compared qualitatively by Kaplan-Meier survival curve and intergroup differences were compared using the log-rank test.

Random Survival Forest (RSF) analysis was used to examine the relative importance of different risk predictors. In RSF, statistical methods are used to estimate the hazard function under the framework of a random forest (8) without making any assumptions about the individual hazard function (9), and ranks the significance of predictors for spontaneous VT/VF. Features and samples are randomly selected for a tree, and log-rank splitting is used to grow the trees. At the end of each branch, a cumulative hazard function is calculated for the selected individual tree. Finally, the ensembled estimated cumulative hazard function is computed by averaging the results of all the trees.

The rfsrc() function of *rfsrc* package and rpart() function of *rpart* package in RStudio (Version 1.1.456) was used to fit a RSF model. Sensitivity analysis on the number of trees and out-of-bag (OOB) prediction performance of the RSF model were then assessed. Survival estimates were calculated using the Brier score (0 = perfect, 1 = poor, and 0.25 = guessing) based on the inverse probability of censoring weight (IPCW) method (10). The cohort was stratified into four groups based on 0–25, 25–50, 50–75, and 75–100 percentile values of incident VT/VF (**Figure 4**).

## Results

### Baseline Characteristics, Genetic Testing, and Pharmacotherapy

This study included 121 consecutive congenital LQTS patients [median age of initial presentation: 20 (interquartile range: 8–44) years, 62% female] with a median follow-up of 88 (51–143) months. The baseline characteristics of the cohort are shown in Table 1. The spontaneous VT/VF incidence rate per 1,000 person-year is 26.2. Family history of LQTS and SCD was present in 39 and 15% of the cohort, respectively. Of the cohort, 69 (52%) and 31 (26%) patients had syncope or spontaneous VT/VF as the initial complaint (of these, 21 patients presented with both syncope and spontaneous VT/VF). EPS studies were rarely conducted (6/121 patients) of which four tested positive. Forty-six (38%) patients underwent 24-h Holter study. Of these, abnormal heart rhythms (sinus arrhythmia, sinus bradycardia, atrioventricular block, progressive cardiac conduction defect, premature atrial complexes, atrial tachycardia or fibrillation, supraventricular arrhythmias, ventricular couplets) were detected in 28 (23%) patients. premature ventricular complexes (PVCs) were seen in 21 (17%) of the patients. Treadmill exercise tolerance test was performed in 40 (33%) patients. ICDs were implanted in 48 (40%) patients.

The article "Territory-Wide Chinese Cohort of Long QT Syndrome: Random Survival Forest and Cox Analyses" was retracted in 2024. Reasons: lack of ethics approval or compliance; concerns about the welfare of human subjects.

**Table 1:** Baseline clinical characteristics and electrocardiographic variables of the included subjects.

**Variable**	**Overall (*n* = 121)**	**VT/VF on follow-up (*n* = 25)**	**No VT/VF on follow-up (*n* = 96)**	***P*-value**
Female gender	76 (62%)	17 (68%)	59 (61%)	0.221
Age of Initial Presentation	20 (8–44)	42 (21–53)	17 (8–37)	**0.003**
Follow-up Period (months)	88 (51–143)	131 (38–163)	85 (51–133)	0.332
Family history of LQTS	47 (39%)	7 (28%)	40 (42%)	0.358
Family history of sudden cardiac death	18 (15%)	2 (8%)	16 (17%)	0.355
Initial presentation with syncope	63 (52%)	18 (72%)	45 (47%)	**0.005**
Syncope	69 (57%)	19 (76%)	50 (52%)	**0.006**
Stress syncope	12 (10%)	2 (8%)	10 (10%)	0.828
Palpitations	22 (18%)	6 (24%)	16 (17%)	0.275
Premature ventricular complexes	21 (17%)	8 (32%)	13 (14%)	**0.014**
Initial presentation with VT/VF	31 (26%)	12 (48%)	19 (20%)	**0.001**
Other arrhythmias^#^	28 (23%)	6 (24%)	22 (23%)	0.710
EPS performed	6 (5%)	3 (12%)	3 (3%)	**0.047**
EPS positive	4 (67%)	1 (33%)	3 (100%)	0.083
Schwartz score	4 (4–5)	5 (4–5)	4 (4–5)	**0.010**
Heart rate	71 (60–92)	69 (59–80)	76 (61–93)	0.300
P-wave duration	102 (93–111)	111 (102–135)	102 (91–110)	0.218
PR interval	158 (146–175)	167 (156–184)	156 (138–172)	**0.029**
QRS duration	90 (84–104)	98 (86–116)	89 (83–100)	0.141
QT interval	447 (402–490)	448 (428–510)	440 (396–482)	0.121
QTc interval	489 (460–516)	493 (467–522)	486 (456–508)	0.380
P-wave axis	61 (37–73)	67 (51–78)	57 (37–72)	0.123
QRS axis	68 (30–83)	60 (20–82)	69 (44–85)	0.360
T-wave axis	53 (23–75)	38 (11–136)	55 (26–73)	0.769
R-wave amplitude in V5	1.07 (0.79–1.52)	1.04 (0.49–1.58)	1.07 (0.82–1.52)	0.739
S-wave amplitude in V1	0.60 (0.38–0.93)	0.60 (0.25–1.54)	0.60 (0.41–0.84)	0.993

# *Other arrhythmias include any brady- or tachy-arrhythmias of non-ventricular origin, sinus node dysfunction and atrio-ventricular block. P-values less than 0.05 are shown in bold text*.

Genetic tests were performed for 61% of the study cohort (Supplementary Table 1). Positive test results, defined as identification of pathogenic, likely pathogenic or variant of uncertain significance if supported by evidence of abnormal ion channel function from functional or clinical studies, were found in 81% of the tested individuals. Five patients had normal genetic tests and the remainder did not undergo testing. The novel mutations not described in cohorts from other geographical regions are marked in Supplementary Table 1. KCNQ1, KCNH2, SCN5A, KCNE1, CACNA1C mutations were identified in 23, 24, 4, 4, and 6 patients, confirming LQTS subtypes 1, 2, 3, 5, and 8, respectively. Single mutations in CAV3 (c.277G>A), AKAP9 (c.6065A>G) and CALM3 (c.286G>C) were found, which corresponded to LQTS types 9, 11 and 16.

The article "Territory-Wide Chinese Cohort of Long QT Syndrome: Random Survival Forest and Cox Analyses" was retracted in 2024. Reasons: lack of ethics approval or compliance; concerns about the welfare of human subjects.

The following six patients had compound mutations. The first had c.782A>G in KCNQ2 and c.328G>A in SCN3B. The latter has been described in a Japanese cohort of Brugada Syndrome (11). However, our patient did not have any Brugada pattern on the ECG. The second patient had the c.31G>A mutation in KCNQ1 and c.56T>C KCNH2. The third patient had the c. 1046C>G mutation in KCNQ1 and c.253G>A mutation in KCNE1. The fourth patient had a variant of uncertain significance and a low clinical significance variant in SCN10A. She had recurrent syncope with ICD implantation but no VT/VF. The final two patients are siblings whose mother died of SCD, with c.1186G>C mutation in CACNAC1 (pathogenic) and c.1627G>A mutation in ANK2 (variant of uncertain significance).

In terms of pharmacotherapy, 107 patients (79.9%) were administered beta-adrenergic receptor blockers. Amongst the 107 patients, the following beta-adrenergic receptor blockers (most common dosage, daily dose) were prescribed: (1) atenolol (*n* = 29, 225 ± 452 mg); (2) bisoprolol (*n* = 8, 1.22 ± 1.37 mg); (3) carvedilol (*n* = 4, 12.9 ± 11.9 mg); (4) labetalol (*n* = 1, 600 ± 0 mg); (5) metoprolol (*n* = 55, 112 ± 89.6 mg); (6) nadolol (*n* = 19, 229 ± 915 mg); (7) nebivolol (*n* = 2, 5 ± 0 mg); (8) propranolol (*n* = 46, 43.1 ± 27.2 mg); sotalol (*n* = 1, 160 ± 0 mg). Mexiletine was prescribed to 12 of the 107 patients (364 ± 113 mg).

### Follow-Up and Predictors of Spontaneous VT/VF Outcomes Post-diagnosis

In total, 23 patients developed VT/VF during follow-up. Kaplan-Meier curves demonstrating freedom from spontaneous VT/VF stratified by age ≥19 years old, PVC, initial presentation with syncope or VT/VF status are shown in Figure 1 (*top left, top right, bottom left and bottom panels*). Significant differences were found between all groups by the log-rank test (*P* = 0.002, *P* = 0.011, *P* = 0.004 and *P* = 0.001, respectively).

The article "Territory-Wide Chinese Cohort of Long QT Syndrome: Random Survival Forest and Cox Analyses" was retracted in 2024. Reasons: lack of ethics approval or compliance; concerns about the welfare of human subjects.

**Figure 1:** Kaplan-Meier survival curves demonstrating freedom from spontaneous ventricular tachycardia/ventricular fibrillation (VT/VF) during follow-up stratified by age ≥19 years of age (top **left**), PVC (top **right**), initial presentation with syncope (bottom **left**), initial presentation with VT/VF (bottom **right**). All showed significant difference between the two groups by the log-rank test.

Univariate Cox regression analysis was performed (Table 2A), revealing that age [hazard ratio (HR): 1.02 (1.01–1.04), *P* = 0.007; optimum cut-off: 19 years], presentation with syncope [HR: 3.86 (1.43–10.42), *P* = 0.008] or VT/VF [HR: 3.68 (1.62–8.37), *P* = 0.002] and the presence of PVCs [HR: 2.89 (1.22–6.83), *P* = 0.015] were significant predictors of spontaneous VT/VF. Only initial presentation with syncope remained significant after multivariate adjustment [HR: 3.58 (1.32–9.71), *P* = 0.011; Table 2B].

**Table 2A:** Univariate Cox regression analysis for shorter time to VT/VF post-diagnosis.

**Variable**	**Hazard ratio (HR)**	**95% confidence intervals (CIs)**	***P*-value**
Female gender	1.53	0.60–3.90	0.372
Age	1.02	1.01–1.04	**0.007**
Initial QTc interval	1.08	1.00–1.02	0.107
Family history of LQTS	0.59	0.24–1.45	0.252
Family history of sudden cardiac death	0.63	0.15–2.71	0.537
Family history of LQTS or SCD	0.61	0.26–1.44	0.261
Initial presentation with syncope	3.86	1.43–10.42	**0.008**
Syncope	4.21	1.43–12.45	**0.009**
Stress syncope	0.76	0.18–3.23	0.705
Palpitations	1.60	0.63–4.07	0.323
Premature ventricular complexes	2.89	1.22–6.83	**0.015**
Initial presentation with VT/VF	3.68	1.62–8.37	**0.002**
Other arrhythmias	0.92	0.36–2.35	0.869
EPS performed	3.77	1.10–12.87	**0.034**
EPS positive	–	–	–
Schwartz score	1.39	0.88–2.21	0.157
Heart rate	0.99	0.97–1.01	0.398
P-wave duration	1.01	0.96–1.05	0.819
PR interval	1.01	0.995–1.031	0.149
QRS	1.01	0.997–1.028	0.104
QT interval	1.01	0.998–1.012	0.128
QTc interval	1.00	0.995–1.012	0.382
P-wave axis	1.00	0.99–1.01	0.857
QRS axis	1.00	0.99–1.01	0.921
T-wave axis	1.00	0.99–1.01	0.936
R-wave amplitude in V5	0.76	0.33–1.76	0.523
S-wave amplitude in V1	1.30	0.37–4.56	0.679

*P-values less than 0.05 are shown in bold text*.

**Table 2B:** Multivariate Cox regression analysis for shorter time to VT/VF post-diagnosis.

**Variable**	**Hazard ratio (HR)**	**95% confidence intervals (CIs)**	***P*-value**
Age	1.02	0.998–1.04	0.073
Initial presentation with syncope	3.58	1.32–9.71	**0.011**
Initial presentation with VT/VF	2.22	0.87–5.64	0.093
Premature ventricular complexes	2.00	0.77–5.21	0.156

*P-values less than 0.05 are shown in bold text*.

The article "Territory-Wide Chinese Cohort of Long QT Syndrome: Random Survival Forest and Cox Analyses" was retracted in 2024. Reasons: lack of ethics approval or compliance; concerns about the welfare of human subjects.

### Random Survival Forest (RSF) Analysis and Comparisons With Cox Proportional Hazard Model

Next, RSF analysis was applied to the present dataset. The data input into the model and relative importance values of the included variables for outcome prediction are shown in Table 3. Sensitivity analysis based on tree number in the RSF model and the derived variable importance ranking were also obtained (Figure 2, *left panel and right panel*). The prediction error becomes smaller when the number of trees in the RSF model increases, indicating that the model learns better when the forest structure becomes more complex. However, this is offset by the disadvantage that more trees take more time for model training and potentially lead to over-fitting. The sensitivity analysis provides a guidance for choosing the optimum number of trees to yield an acceptable prediction error without overcomplicating the model. Marginal effects reveal how a dependent outcome variable varies when the independent variable changes. The survival curve and cumulative hazard function generated by the RSF model is detailed in Figure 3 (*left panel and right panel*).

**Table 3:** Variable importance ranking to predict VT/VF post-diagnosis with RSM model.

	**Importance**	**Relative importance**
Age	0.0815	1.0000
Schwartz score	0.0057	0.0705
Family LQTS	0.0035	0.0427
Sex	0.0022	0.0269
Family SCD	0.0018	0.0223
Initial QTc interval	−0.0030	−0.0369
Other arrhythmias	−0.0045	−0.0551
Initial VT/VF	−0.0091	−0.1120

**Figure 2:** Optimal tree number selection (**Left**) and variable importance ranking for RSF model to predict VT/VF in LQTS (**Right**).

**Figure 3:** Predicted OOB survival (**Left**) and cumulative hazard (**Right**) curves generated from the RSF model to predict VT/VF post-diagnosis.

Survival estimates from the RSF model are shown in Figure 4. A survival function was determined for each LQTS patient. In the top left panel, the red line illustrates the overall ensemble survival, whereas the green line shows the Nelson-Aalen estimator. The top right panel shows Brier score (0 = perfect, 1 = poor, and 0.25 = guessing) stratified by ensemble spontaneous VT/VF based on the inverse probability of censoring weight (IPCW) method (10). The cohort was stratified into four groups of 0–25, 25–50, 50–75, and 75–100 percentile for the occurrence of spontaneous VT/VF (the overall non-stratified Brier score is shown by the red line). The bottom left panel shows the continuous rank probability score (CRPS) given by the integrated Brier score divided by time, whereas the bottom right panel shows a plot of VT/VF postdiagnosis of each patient against time.

The article "Territory-Wide Chinese Cohort of Long QT Syndrome: Random Survival Forest and Cox Analyses" was retracted in 2024. Reasons: lack of ethics approval or compliance; concerns about the welfare of human subjects.

**Figure 4:** Survival estimates. Survival function estimated for each LQTS patient from the random survival forest (RSF) model (overall ensemble survival is indicated by the red line; the Nelson-Aalen estimator is given by the green line) (top **left**). Brier score (0 = perfect, 1 = poor, and 0.25 = guessing) stratified by ensemble spontaneous VT/VF based on the inverse probability of censoring weight (IPCW) method (top **right**). The cohort was stratified into four groups of 0–25, 25–50, 50–75, and 75–100 percentile spontaneous VT/VF (the overall, non-stratified, Brier score is shown by the red line). Continuous rank probability score (CRPS) given by the integrated Brier score divided by time (bottom **left**). Plot of spontaneous VT/VF of each LQTS patient against time (bottom **right**). Events are shown as blue points, whereas censored observations are shown as black points.

Finally, comparative analysis showed that the RSF model showed an improved performance compared to Cox regression model as illustrated by the higher values in precision, recall, AUC and Harrell's C index with a 5-fold cross validation approach (Table 4). Decision rules were generated by RSF model to predict VT/VF post-diagnosis as shown in Figure 5. ROC and AUC of RSF model to predict VT/VF post-diagnosis were presented in Figure 6.

**Table 4:** Performance comparisons of RSF and multivariate Cox models to predict VT/VF post diagnosis with 2-fold cross validation approach.

**Model**	**Precision**	**Recall**	**Brier score**	**AUC**	**Harrell's C index**
RSF	0.80	0.79	0.10	0.77	0.79
Multivariate Cox	0.69	0.68	0.16	0.68	0.67

**Figure 5:** Decision rules generated by RSF model to predict VT/VF post-diagnosis.

**Figure 6:** ROC and AUC of RSF model to predict VT/VF post-diagnosis.

## Discussion

In this territory-wide study of congenital LQTS patients, the main findings are: (i) the identification of novel mutations in a number of putative ion channel genes, (ii) family history of LQTS or SCD, initial presentation with syncope or VT/VF, the presence of PVCs, QTc interval and QRS duration were significant predictors of spontaneous VT/VF on univariate Cox regression and only prior presentation with VT/VF remained significant after multivariate adjustment; (iii) RSF model provided significant improvement in risk prediction over Cox regression.

### Genetic Heterogeneity in a Chinese Cohort of Congenital LQTS

Loss-of-function mutations in various potassium channel subunits are responsible for LQTS types 1 (KCNQ1), 2 (KCNH2), 5 (KCNE1), 6 (KCNE2), 7 (KCNJ2), and 13 (KCNJ5). Gain-of-function mutations in sodium channel subunits lead to LQTS types 3 (SCN5A) and 10 (SCN4B), and in the L-type calcium channel produces LQT type 8 (CACNA1C, Timothy syndrome). Mutations in supporting proteins are responsible for the LQT type 4 (ANKB), 9 (CAV3), 11 (AKAP9), and 12 (SNTA1) phenotypes. The underlying mechanisms can be due to a direct reduction in gating properties, or altered expression, localization or trafficking of these ion channel proteins affecting repolarization or late depolarization. Genetic analysis identified novel mutations in KCNQ1, KCNH2, SCN5A, ANK2, CACNA1C, CAV3, AKAP9, and HCN4.

The article "Territory-Wide Chinese Cohort of Long QT Syndrome: Random Survival Forest and Cox Analyses" was retracted in 2024. Reasons: lack of ethics approval or compliance; concerns about the welfare of human subjects.

The following novel mutations in KCNQ1 were identified. The c.31G>A mutation in exon 1 leads to E11K variant, altering the secondary structure of this subunit. *In silico* analysis predicts this mutation to be probably damaging to channel function. The Human Gene Mutation Database has reported two mutations in nearby regions, A2V, P7S, in the context of LQTS (12). The c.782A>G mutation in exon 6 affects the S4/S5 region and is predicted to be likely pathogenic. The c.1018T>C mutation in exon 7 affecting the S5-pore-S6 region and c.1831G>A in exon 16 affecting the C-terminus are pathogenic. Three novel KCNH2 mutations were found. Firstly, c.211G>T in exon 2 affecting the N-terminus is pathogenic. A different missense variant affecting the same codon, c.211G>C has been reported previously in LQTS patients (13, 14). The c.1738G>A in exon 7 affects the S5-pore-S6 region. The c.1738G>C mutation affecting the same codon was reported to be likely pathogenic (VCV000191223.1).

The c.1627G>A mutation in ANK2 leads to a change in amino acid from valine to methionine in the membrane-binding domain and has not been described in LQTS. It has been classified as a variant of uncertain significance, but the valine is located at a moderately conserved region (VCV000526909.1). In the two siblings harboring this mutation, the pathogenic variant c.1186G>C in CACNA1C was also found. It was therefore not possible to examine the relative contributions of these variants to the electrophysiological phenotype.

Moreover, a mutation in CAV3, c.277G>A leading to p.Ala92Thr, was identified in a neonatal patient who presented with supraventricular tachycardia associated with prolonged QTc of values between 450 and 480 ms. CAV3 encodes for the scaffolding protein caveolin-3, which is the main component of caveolae. Previously, autosomal recessive c.277G>A mutation was associated with rippling electromyographic discharges with muscular dystrophy (15), whereas heterozygotes were asymptomatic with normal cardiac function but electrocardiographic findings were not reported (16). Nevertheless, the p.Ala85Thr and p.Phe97Cys mutations were linked to a persistent late sodium current in LQTS (17). Given that caveolin-3 and the SCN5A subunit co-localize in the cell membrane, the CAV3 mutation in our patient may increase the QTc interval by increasing the late sodium current, but this remains to be elucidated in functional studies.

The article "Territory-Wide Chinese Cohort of Long QT Syndrome: Random Survival Forest and Cox Analyses" was retracted in 2024. Reasons: lack of ethics approval or compliance; concerns about the welfare of human subjects.

A mutation in AKAP9 was detected in an asymptomatic young boy with ECG findings of QTc prolongation to 485 ms, slow rising T-waves, T-wave inversion in V1–V3 and notched waves in V4–V6. He initially presented with seizures and had a diagnosis of XL creatine transporter deficiency. AKAP9 encodes for the kinase-anchor protein-9 and is recognized as a genetic modifier of congenital LQTS (18). Its loss-of-function mutations have been associated with congenital LQTS type 11 (19).

In addition to the novel mutations described above, our study also identified pathogenic variants in KCNQ1, KCNH2, SCN5A, and KCNE1. Moreover, the D96V mutation in CALM3 (c.286G>C leading to p.Asp96His) was also found in one patient. This mutation was previously associated with severe QTc prolongation to 690 ms with 2:1 atrioventricular block and T-wave alternans, recurrent VF and aborted SCD events accompanying cerebral seizures (20).

### Mechanisms of Ventricular Arrhythmogenesis in Congenital LQTS

Univariate Cox regression findings using clinical electrocardiographic data demonstrate that PVCs and prolonged QTc intervals predicted incident spontaneous VT/VF. They therefore support the trigger-substrate hypothesis in LQTS (21). Significant predictors of spontaneous VT/VF were syncope at initial presentation or occurring at follow-up. in accordance findings from previous studies investigating congenital LQTS cohorts (22, 23). Family history of LQTS was identified as a protective factor. The reason is that family members of the probands who were tested positive for the genetic mutations, but without spontaneous VT/VF events, were also included. As many were silent carriers, their inclusion meant that the hazard ratios were skewed to lower values.

### Improved Prediction of Spontaneous VT/VF Using Random Forest Analysis Compared to Cox Regression

RSF builds hundreds of trees and generates outcome prediction by voting method for analyzing right censored survival data (8). The advantage is that unlike the Cox proportional hazard model, it does not make assumptions about the individual hazard function (9) and ranks the significance of predictors for spontaneous VT/VF. Randomization is introduced in two forms: a randomly drawn bootstrap sample of data for growing the tree, and nodes splitting on randomly selected predictors for growing the tree learner. The boosting tree structure in RSF can capture the nonlinear effects and complex interactions among the variables, which can reduce prediction variance and bias as well as significantly improve learning performance (9). Moreover, RSF can handle the effects of the treatments and predictor variables, whereas traditional methods using Cox or Kaplan Meier analysis utilize a linear combination of attributes (24). RSF has been applied to improve prediction of all-cause mortality, heart failure-related hospitalizations, cost and home days loss in heart failure (25) in addition to mortality prediction in heart failure patients undergoing cardiac resynchronization therapy (26). Moreover, it successfully predicted inpatient mortality following cardiac arrest after admission to intensive care (27), sudden cardiac arrest in the Left Ventricular Structural (LV) Predictors of Sudden Cardiac Death (SCD) Registry (28) and all-cause mortality prediction in acquired long QT syndrome (29). Our study demonstrates for the first time that RSF model can significantly improve spontaneous VT/VF prediction in inherited LQTS.

The article "Territory-Wide Chinese Cohort of Long QT Syndrome: Random Survival Forest and Cox Analyses" was retracted in 2024. Reasons: lack of ethics approval or compliance; concerns about the welfare of human subjects.

## Limitations

Several limitations should be noted. Firstly, this was a retrospective study. Nevertheless, for most patients, six-monthly to annual follow-ups were available. In Hong Kong, all public hospitals have linked electronic health records, meaning that if patients are admitted to another hospital, the case records and investigation results can be traced back and viewed electronically. Secondly, the predictive value of investigations was limited by the relatively small sample size of this cohort. Thirdly, only scanned ECGs were available and therefore the ECG variables summarized were averaged from the 12 leads. The raw ECG files could not be obtained and therefore it was not possible to extract the measurement from each lead. Future work should explore the possibility of converting scanned images to electronic ECG files for detailed analyses, for example to investigate whether the incorporation of novel indices such as T-wave morphology can further enhance diagnosis or risk prediction (30, 31). Fourthly, for some patients, only Sanger sequencing of targeted genes was performed, without next generation sequencing (NGS) of their entire genomes. Therefore, contributions from mutations in other genes cannot be excluded. Because genetic tests were not performed in all of the LQTS patients included, our risk model did not include genetic results as a predictive variable. Other studies have reported that genotype is an important determinant of arrhythmic risk (32–34), and prospective studies should be conducted to identify genetic risk factors. Finally, the family history of LQTS was low because the medical records for the relatives of probands were often not accessible, unless the attending physicians specifically noted down the identity details or coded them with ICD-9 codes.

The article "Territory-Wide Chinese Cohort of Long QT Syndrome: Random Survival Forest and Cox Analyses" was retracted in 2024. Reasons: lack of ethics approval or compliance; concerns about the welfare of human subjects.

## Conclusions

Effective risk stratification in congenital LQTS can be achieved by clinical history, electrocardiographic indices, and different investigation results, irrespective of underlying genetic defects. A machine learning approach using RSF can improve risk prediction over traditional Cox regression models.

## Data Availability Statement

The datasets presented in this study can be found in online repositories. The names of the repository/repositories and accession number(s) can be found below: https://doi.org/10.5281/zenodo.3465850, Zenodo.

## Ethics Statement

The studies involving human participants were reviewed and approved by The Joint Chinese University of Hong Kong–New Territories East Cluster Clinical Research Ethics Committee. Written informed consent from the participants' legal guardian/next of kin was not required to participate in this study in accordance with the national legislation and the institutional requirements.

## Author Contributions

GT, SL, and JZ: data collection, clinical data analysis, manuscript drafting, and manuscript critical revision. TL and IW: data analysis and manuscript critical revision. CM, NM, and KJ: data collection, genetic analysis and interpretation, ECG analysis, and manuscript critical revision. QZ, SC, and WTW: genetic results interpretation, manuscript critical revision, and study supervision. All authors contributed to the article and approved the submitted version.

## Conflict of Interest

The authors declare that the research was conducted in the absence of any commercial or financial relationships that could be construed as a potential conflict of interest.
